The article "A Face Recognition System Using ACO-BPNN Model for Optimizing the Teaching Management System" was retracted in 2023. Reasons: suspected computer-generated content; unreliable results or conclusions; concerns about the data; concerns about the results or conclusions.

# A Face Recognition System Using ACO-BPNN Model for Optimizing the Teaching Management System

**DOI:** 10.1155/2021/5194044

**Published:** 2021-09-02

**Authors:** Xiuli Zhu

**Affiliations:** ^1^School of Education Science and Psychology Science, Chengdu Normal University, Sichuan, Chengdu 611130, China; ^2^School of Educational Sciences, Nanjing Normal University, Jiangsu, Nanjing 210097, China

## Abstract

The basic idea of face recognition technology is to compare the matching degree between the standard face image marked with identity information and the static or dynamic face collected from the actual scene, which includes two main research contents: face feature extraction and face feature recognition. Traditional identification generally proves who we are through certificates, passwords, or certificates plus passwords. With the development of science and technology, face recognition technology will occupy an increasingly important position. Inspired by the human brain, the artificial neural network (ANN) is an information extraction system based on imitating the basic function and structure of the human brain and abstracted by physical and mathematical research methods. Based on the traditional BP neural network model, this paper proposes an ant colony algorithm-enabled BP neural network (ACO-BPNN) model and applies it to face recognition. Experimental results show that, similar to other face recognition techniques, the facial feature location needs to adapt to various changes of faces to the maximum extent, so the recognition and classification effect of the whole face feature extracted from the whole face image on the changes of such partial areas is not good, while the local feature extraction method based on ACO-BPNN can achieve a good recognition and classification effect.

## 1. Introduction

In recent decades, neural computing with neural networks as the research object has developed rapidly as a practical technology and has been successfully applied in many fields, including the field of school education and teaching management which is one of the main and most successful applications is pattern recognition [1]. In fact, it is a dynamic mathematical model with a directed graph as the topological structure, which realizes distributed parallel processing of continuous or discrete inputs by adjusting parameters, which is also called a neural network algorithm. Traditional identification generally proves who we are through certificates, passwords, or certificate plus passwords. We all know these traditional identification methods. Everyone often uses them, but they also bring many hidden dangers [2]. The face recognition rate is one of the indicators for judging the performance of face recognition technology. In order to improve the recognition rate, artificial neural network technology can be used to complete facial image recognition [3]. In order to simulate the thinking mode of human brain, we need to understand the biology of the human brain. After optimization, the ant colony neural network strengthens many minimal problems and improves the previous problems such as slow speed [4].

Face recognition has been widely used in the human-computer interface because of its good interaction [5]. The basic idea of face recognition technology is to compare the matching degree between the standard face image with the identified information and the static or dynamic face collected from the actual scene, which includes two main research contents: face feature extraction and face feature recognition. But the previous face recognition system is not perfect, and its practical application is significantly poor. This is also the aspect that we should improve in the later period. For example, identity information theft is a common problem in all over the world, and the amount of loss is heavy. With the convenience and high efficiency of the network, face recognition technology will be popularized [6]. The distribution of the various organs of the face is similar, and the appearance of the organs of the face is very similar, and the individual difference is not large. This feature is not good for the face recognition classification [7]. In addition, face images are volatile. The facial expressions, different image acquisition angles, different lighting conditions, and face coverings (glasses, masks, etc.) will all bring great differences to the same face [8]. Therefore, improving the recognition accuracy of the face recognition system under complex conditions is a problem we need to study and improve. This is also a problem that must be solved to optimize the teaching management system with face recognition technology.

Inspired by the human brain, the artificial neural network (ANN) is a kind of information output system based on imitating the basic functions and structures of the human brain and abstracted by physical and mathematical research methods [9]. Compared with the above problems, the advantages of the face recognition method based on the neural network are also very prominent, such as (1) avoiding the manual design of feature extraction methods. (2) Its parallel processing of information is more conducive to using hardware to improve the recognition speed. (3) As one of the key technologies of artificial intelligence, it is possible to make the machine have the same face recognition ability as human beings or even surpass human beings [10]. At present, various countries have launched special research groups based on this aspect [11]. Zhang et al. have also carried out research on face recognition [12]. There are few research studies on optimizing the teaching management system with face recognition technology based on the neural network. To sum up, this paper proposes an ant colony algorithm-enabled BP neural network (ACO-BPNN) model for the teaching management system in face recognition.

## 2. Related Work

Face recognition with a computer cannot be completed in one step, and it requires many steps. Generally, this is called a face recognition system and refers to the software part that realizes face recognition. Cho and Jeong [13] proposed a semiautomatic face recognition system model and feature extraction method, which aroused the interest of many practitioners, experts, and scholars, and it has also aroused the interest of the school teaching management reform personnel and researchers. Ozyurt and Ozyurt [14] summarized the biological structure, function, and working principle of neuron cells and realized neuron cells with mathematical model abstract simulation. This model is the M-Р model. Yin and Liu [15] proposed that when the data samples are linearly inseparable, the support vector machine uses the so-called “core mechanism” nonlinear mapping algorithm to transform the linearly inseparable samples into a high-dimensional feature space to make them linearly separable. The core of the algorithm in [16] used the so-called “restricted Boltzmann machine” to learn from Boltzmann's thought. RBM is a two-layer network, which can be used for “unsupervised training” of neural networks. Yang et al. [17] put forward a famous perceptron model, which is a neural network model with the three-layer structure, which is composed of many threshold neuron cell models connected by hierarchical topology. By learning and training to change the weight of connection, different models can be classified correctly. Long et al. [18] trained the neural network system with nearly 10,000 handwritten digit samples provided by the US Postal System, and the error rate in independent test samples is as low as 5%, reaching the practical level.

In order to solve the problem of overfitting, a new algorithm called “discard” is proposed in [19]. The purpose of the discarding algorithm is to give each neuron a certain probability in each training, assuming that it does not exist and not to add it when calculating. Hao [20] used an excitation function called “modified linear element” in the algorithm of this paper. Compared with using other excitation functions, the error rate of “corrected linear unit” will be lower. The so-called “sparse representation” is formed naturally, which can express abstract and complex concepts efficiently, flexibly, and robustly with a small number of neurons. Shao and Guo [21] officially put forward the use of the reverse algorithm so that the error correction calculation is reduced to a state equal to the number of neurons only. Feng and Chen [22] put forward the theory that the strength of the synapses connected between neuron cells is variable. It is believed that if both the original neuron cell and the target neuron cell are activated, the axon and dendrites between them are the connection strength will be strengthened. Han et al. [23] simply discussed that when the function propagates back from the output layer, the gradient decreases rapidly, but the learning speed becomes extremely slow every time it passes through the output layer. The neural network can easily stagnate in the local optimal deep learning solution.

## 3. Methodology

### 3.1. Introduction to Face Recognition Technology

As early as the early days of computer vision research in 1960s and 1970s, face recognition aroused strong interest of researchers. Traditional neural network face recognition must be combined with some artificially designed feature extraction algorithms, and face features can only be classified and recognized after being digitized [24]. Its learning is more inclined to the classification of face feature vectors, and neural networks are all shallow, that is, networks with fewer layers [25]. It is a system which is interconnected by many very simple processing units working in parallel in a certain way and dynamically responds to external input signals. However, the deep learning method improves the ability of the neural network by deepening and increasing the neural network structure [26]. And, the focus of network learning is transferred from feature classification to feature extraction. In the early 1970s, the United States, the United Kingdom, Japan, Canada, and other countries began the work of face recognition and achieved a certain degree of development [27]. Secondly, at that time, the computing power was too low to support the amount of computation required by the neural network model. So far, the research of the neural network has been extended to automatic driving, robot, machine vision, natural language processing, pattern recognition, image classification, school education activities, teaching management, as well as teacher management, student management, and other fields related to artificial intelligence. Especially, in the aspect of face recognition, people have started the related research for a long time.

Specific operation of face recognition: first obtain the face image through the image acquisition device, and preprocess the image. Detect the processed image to detect whether there is a human face in the image [28]. If it exists, locate the face position and obtain the face information required for face recognition. Face recognition needs to be screened layer by layer, which is complicated that we cannot feel intuitively. Here, we need to identify our facial features, so as to clearly understand your features. The features extracted from the training samples are trained into a library, and the same method is used to obtain the features extracted from the sample to be tested. Match this feature with the features in the face database [29]. If there is a matching feature, the identity of the sample to be tested can be obtained. Through face data, researchers can verify the new algorithm or improve the existing algorithm to improve the accuracy of face recognition. The function it can achieve is relatively simple, and the intelligence it can achieve is also very simple, which cannot be compared with human brain thinking, but this simple model can show some skill characteristics of the brain thinking mode, such as learning ability, self-adapting ability, and self-organizing ability. Finally, face recognition compares the features and data with the current face database to verify the identity.

At present, many existing multipose face recognition algorithms are tested and optimized on the face database. Because the collected face images are affected by various interference factors, such as light, shadow, occlusion, and collection angle, therefore it is necessary to process the face feature data after interference. After preprocessing, high-quality sample feature data can be obtained. The main purpose of classification and recognition is to match the features of the images to be recognized with the features of the images in the database. There are two main tasks of recognition. One is face recognition, which uses the currently recognized face to compare and search in the database [30]. This is a one-to-many matching process. The second is face verification, which is a one-to-one matching process.

### 3.2. The Proposed ACO-BPNN Model

Each neuron cell is composed of an axon and a plurality of dendrites, and each neuron cell is connected with axons of a plurality of neuron cells through a plurality of dendrites and used for receiving stimulation signals. The artificial neural network (ANN) is a nonlinear dynamic system with good adaptability and wide application range [31–37], especially in pattern recognition. In order to improve the adaptive performance of the face recognition system, we proposed the ACO-BPNN model, as shown in Figure 1.

ACO-BPNN is a simulated evolutionary algorithm. Preliminary research shows that the algorithm has many excellent properties.

The main steps of ACO-BPNN model training neural network weights and thresholds are as follows:

(1) Set the initial conditions: let time *t*=0 and *NC*=0 iterations, set the maximum number of iterations *NC*_max_, the number of ants *K*, let the pheromone *τ*_*j*_(*I*_*pi*_)〈0〉=*C*(0) of element *j* in *I*_*pi*_ (1 ≤ *I* ≤ *m*), and Δ_*τ*_*j*__(*I*_*pi*_)=0, and put all ants in the nest.
(2) Start all ants, each ant *k* starts from the first set, and selects an element in each set in turn according to the following rules. Path selection rule: for set *I*_*pi*_, any ant *k*(*k*=1,2,…, *K*), randomly select its *j*th element according to the probability calculated by the following formula [29]:
  (1) $$\begin{array}{c} P\left(\tau_{j}^{k}\left(I_{pi}\right)\right)=\frac{\tau_{j}\left(I_{pi}\right)}{\sum_{\mu =1}^{N}\tau_{u}\left(I_{pi}\right)}, \end{array}$$
until all the ant colonies reach the food source.
(3) When all ants select an element in each set and return to the nest according to the original path, the pheromone of the selected element will be adjusted according to the following formula if the time of the process is *n* time units.

(2) $$\begin{array}{c} \tau \left(I_{pi}\right)\left(t+n\right)=\rho c_{j}\left(I_{\left.pi\right)}\left(t\right)+\Delta \tau_{j}\left(I_{pi}^{}\right.\right),\\ \Delta \tau_{j}\left(I_{pi}\right)=\sum_{k=1}^{k}\Delta \tau_{j}^{k}\left(I_{pi}\right). \end{array}$$

Among them, the parameter *ρ*(0 < *ρ* < 1) represents the persistence of the pheromone, 1 − *ρ* represents the degree of pheromone disappearance, and Δ*τ*_*j*_^*k*^(*I*_*pi*_) represents the pheromone left by the *k*th ant on the *j*th element of the set *I*_*pi*_ in this cycle, which can be calculated by the following formula:

(3) $$\begin{array}{c} \Delta \tau_{j}^{k}\left(I_{pi}\right)=\left\{{}_{0}^{Q/e_{k}}|.\right. \end{array}$$

In equation (3), *q* is a constant for adjusting the speed of pheromone adjustment and *e*_*k*_ is an output error, *e*_*k*_=*O*_*n*_ − *O*_*q*_, which takes a set of weights and thresholds selected by the *k*th ant as weights and thresholds of the neural network, where *O*_*n*_ and *O*_*q*_ are the actual and expected outputs of the neural network. The smaller the error, the more the corresponding pheromones increase.

Repeat the above steps until all ants converge to a path or reach the maximum number of iterations *NC*_max_ and output the optimal solution.

By selecting the sample image data of 10 people, the training sample and the test sample are taken from the sample image data, and each person is trained with 10 images and tested with 4 images. The traditional BP neural network classifier and the ant colony optimization BP neural network classifier are used for classification, respectively. Compare the recognition rate of the ant colony optimization BP neural network and BP neural network, as shown in Figure 2.

The basic idea of ACO-BPNN training neural network weights and thresholds is suppose there are M parameters in the network, including all weights and thresholds. Even if the input information is incomplete, inaccurate or ambiguous, the ACO-BPNN model can still associate the complete image of the things in the memory. The ACO-BPNN algorithm is a mathematical modeling and simulation of the operation process of the biological neural network in the human brain, which is composed of a large number of highly interconnected biological neurons. Therefore, the ACO-BPNN algorithm can also be regarded as the artificial neural network, which is formed by connecting mathematical models of biological neurons. ACO-BPNN is composed of several parallel computing neurons connected by the neuron layer. With the development of science and technology and the continuous enhancement of computer computing capabilities, artificial neural networks have the characteristics of adaptive learning, robustness and fault tolerance, distributed parallel processing, and nonlinear mapping.

Because of the simple connection of artificial neurons, the network implies some kind of the similar human brain, such as learning, generalization, adaptation, fault tolerance, and distributed representation. The traditional BP network adopts the gradient descent algorithm in the learning process, which has the problems of slow convergence, turbulence in the training process, and easy to fall into a local minimum. In order to reduce the vibration in the training process, a momentum term can be introduced to reflect the accumulation of previous experience of weights.

The relationship between the number of feature vectors selected when using traditional BP neural network as the classifier and ACO-BPNN as the classifier and the recognition rate of test images, as shown in Figure 3.

The weight adjustment of the BP network is not only related to the gradient of error term to weight but also related to the previous weight adjustment. The weight adjustment formula is as follows [21]:

(4) $$\begin{array}{c} \Delta W\left(t+1\right)=\left(1-mc\right)\eta \delta x+mc\Delta W\left(t\right). \end{array}$$

Among them, Δ*W*(*t*) is the change of the weight, *t* is the number of training, the momentum coefficient is represented by *mc*, *η* is the learning rate, *δ* is the error term, *x* is the input, and *δx* essentially reflects the gradient of the error term to the weight. It can be seen that the additional momentum method takes into account the influence of the accumulation of previous experience on the adjustment of the weight, and the momentum coefficient is *mc* ∈ (0,1). The relationship between the size of the weight adjustment and the update value is

(5) $$\begin{array}{c} \Delta W\left(t\right)=\left\{\begin{array}{cc} -\Delta t, & \frac{\partial E\left(t\right)}{\partial W}>0,\\ +\Delta t, & \frac{\partial E\left(t\right)}{\partial W}<0,\\ 0, & \frac{\partial E\left(t\right)}{\partial W}=0. \end{array}\right. \end{array}$$

Then, the corresponding weight adjustment formula at time *t* + 1 is

(6) $$\begin{array}{c} W\left(t+1\right)=W\left(t\right)+\Delta W\left(t\right). \end{array}$$

The adjustment rule of update value Δ*t* is as follows:

(7) $$\begin{array}{c} \Delta t=\left\{\begin{array}{cc} \alpha \times \Delta \left(t-1\right), & \frac{\partial E\left(t\right)}{\partial W}\times \frac{\partial E\left(t-1\right)}{\partial W}>0,\\ \beta \times \Delta \left(t-1\right), & \frac{\partial E\left(t\right)}{\partial W}\times \frac{\partial E\left(t-1\right)}{\partial W}<0,\\ \Delta \left(t-1\right), & \frac{\partial E\left(t\right)}{\partial W}\times \frac{\partial E\left(t-1\right)}{\partial W}=0. \end{array}\right. \end{array}$$

Among them, 0 < *β* < 1 <*α*.

When the scale of the histogram feature is 8, 20, and 30, the corresponding recognition performance curve of the face recognition algorithm is obtained, as shown in Figure 4.

By introducing the elastic gradient descent method, the adverse effect of the gradient on the network is overcome, and the network can converge quickly.

## 4. Result Analysis and Discussion

### 4.1. Overview of Face Recognition under Complex Lighting Conditions

Face recognition is a typical subject in the field of pattern recognition and image analysis. As an authentication technology, face recognition technology is widely used in finance, security, and other fields. It is urgent to introduce this technology into the field of school education, especially in the field of teaching management, so as to improve its efficiency and the quality of education. The face images we get under different illumination conditions have a great influence on the accuracy of the face recognition system. When this part of the reflected or transmitted light enters the camera, it is converted into a digital array of gray or color values in the imaging plane, which produces the image. However, under the influence of different illumination, different collection angles, and different expressions, the facial features of the same person will show great differences, which cause great difficulties in face recognition. Under natural conditions, the pose of the human face is diverse, and the face images we capture cannot always be positive. Any small head movement of deflection, looking up or looking down will cause varying degrees of distortion to the expression of face information, as shown in Figure 5.

The features extracted from distorted face images are bound to have a certain impact on the effect of face recognition. In the process of classroom teaching and its management, the light and shadow changes caused by the individual activities and diversified scenes of teachers and students also increase the difficulty of face recognition. The influence of illumination on face recognition is far greater than imagined, and the face images obtained by the same person under different illumination conditions are even more different than those of different people under the same illumination conditions.

Similar to other face analysis techniques, facial feature location needs to adapt to various changes of faces to improve the robustness of the algorithm. Therefore, the recognition and classification effect of the whole face feature extracted from the whole face image on the change of this partial region is not good, but the local feature extraction method can achieve a good recognition and classification effect. Human vision is derived from the response of the human visual system to external light. When light hits the surface of an object, the light may be absorbed, reflected, and transmitted. The main reason is that the human face is nonrigid and is easily affected by factors such as light, posture, and expression. When the face is covered by 10%, the location accuracy of the projection reverse combination algorithm is the worst. When the face is covered by 30%, the projection reverse combination tends to diverge, which means that the face cannot be accurately fitted. The advantage of this algorithm is the most obvious, as shown in Figures 6 and 7.

In addition, with the increase of age, the face will change greatly. The students in the school teaching management, especially the middle and primary school students in the growth peak period, their faces change more greatly. Light also plays a vital role in face recognition because light can directly affect our facial features. This is a great challenge to face recognition. These will significantly affect the description of face features, thus affecting the effect of face recognition. But in practical application, the nonideal shooting environment and the mismatching of image recognition will greatly affect the performance of the system. The face database is used to locate and separate the background of standardized human face images under different lighting conditions.

### 4.2. Face Feature Extraction Method

Face description features can be generally divided into three categories: global features, local features, and global and local fusion features. For example, the change of illumination will cause shadow in the face image, and the change of head posture and expression will change the image shape near the feature points, and the obstacles such as glasses, beard, or arms will make the feature points disappear or deform. In order to recognize faces under complex illumination conditions, the illumination information should be reduced as much as possible in the feature vectors obtained in the feature extraction stage, and more information of the original face images should be retained. In addition, the word “automatic” in the definition of the automatic face recognition system is largely attributed to the automatic completion of face detection. Generally speaking, facial feature points are located at the tip or protruding part of facial features contour, such as inner and outer corners of eyes, corners of mouth, and tip of nose. The recognition rate data recorded during the simulation experiment by changing the wavelet basis function and the wavelet transform layers in turn are shown in Table 1.

It can be seen from the data in the above table that, under the same conditions, the optimal face recognition effect can be obtained by selecting the Daubechies (db3) wavelet basis function for quadratic discrete wavelet transform of the face image. The wavelet function and its scaling function are shown in Figures 8.

However, it is very difficult to locate and track face feature points from video images according to this texture information because feature points are full of changes. Finally, based on the projection inverse combination algorithm, the inverse combination algorithm based on prior knowledge is applied to optimize the energy equation and constraint equation simultaneously. Feature extraction is one of the key technologies in the face recognition system, which refers to the process of describing face features by calculating and analyzing face images to obtain data with certain discrimination. In reality, the process and related environment of teacher management, student management, teacher-student interaction, and teaching management are very complicated. How to find a face description feature that is not affected by the complex environment is one of the most effective methods to solve the problems of lighting, posture, etc. Both global features and local features cannot contain all the information of face, and the development trend of feature extraction in the future will gradually develop in the direction of global and local multifeature fusion.

## 5. Conclusions

Face recognition is an interdisciplinary hot research issue. Because the face is a three-dimensional nonrigid object with expression, posture, and various changes, the uncertain factors such as beard, hairstyle, glasses, and light intensity make the face pattern more complex. Therefore, face recognition is a challenging frontier subject with high academic value and application prospect. The face recognition method based on ACO-BPNN avoids the manual design of the feature extraction method, and its parallel processing of information is more helpful to improve the recognition speed by using hardware. Similar to other face analysis techniques, the face feature location needs to adapt to all kinds of face changes to the greatest extent, so the whole face feature extracted from the whole face image has poor recognition and classification effect on such local area changes, while the local feature extraction method based on ACO-BPNN can achieve good recognition and classification effect. Due to the complexity and variability of illumination, although there are many algorithms to deal with illumination problems at present, the actual results are far from meeting people's requirements. In the future, we still need to continue to study and delve into the knowledge related to face recognition and neural network and strive to advance towards the intelligent research direction of face recognition.

## Figures and Tables

**Figure 1:** The architecture of the ACO-BPNN model.

**Figure 2:** Comparison of the recognition rate between the ACO-BPNN model and BPNN model.

**Figure 3:** The relationship between the recognition rate of the test image and the number of feature vectors.

**Figure 4:** The impact of the feature scale on the recognition rate.

**Figure 5:** Face images of the same person under different lighting.

**Figure 6:** When the face is covered by 10%, the positioning accuracy of the two algorithms.

**Figure 7:** When the face is covered by 30%, the positioning accuracy of the two algorithms.

**Figure 8:** The image of the wavelet function and its scaling function.

**Table 1:** The influence of wavelet basis function and the number of wavelet transform layers.

Wavelet basis function	Haar	Db1	Db2	Db3	Db4	Db5	Db6	Db7
1-layer wavelet basis function	76.8	77.2	80.9	82.1	86.4	89.7	78.7	79.6
2-layer wavelet basis function	62.8	62.1	56.4	76.4	59.6	57.7	64.3	63.9

## Data Availability

The data used to support the findings of this study are available from the corresponding author upon request.

## References

[1] Di C., Peng J., Di Y., Wu S. (2021). 3D face modeling algorithm for film and television animation based on lightweight convolutional neural network. *Complexity*.

[2] Meden B., Mallı R. C., Fabijan S., Ekenel H. K., Štruc V., Peer P. (2017). Face deidentification with generative deep neural networks. *IET Signal Processing*.

[3] Dang L. M., Hassan S. I., Im S., Moon H. (2019). Face image manipulation detection based on a convolutional neural network. *Expert Systems with Applications*.

[4] Alarifi A., Tolba A., Al-Makhadmeh Z., Said W. (2020). A big data approach to sentiment analysis using greedy feature selection with cat swarm optimization-based long short-term memory neural networks. *The Journal of Supercomputing*.

[5] Choi J. Y. (2017). Improved deep face identification with multi‐class pairwise discriminant loss. *Electronics Letters*.

[6] Gavrilescu M. (2016). Study on using individual differences in facial expressions for a face recognition system immune to spoofing attacks. *IET Biometrics*.

[7] Thanga Selvi R., Muthulakshmi I. (2021). An optimal artificial neural network based big data application for heart disease diagnosis and classification model. *Journal of Ambient Intelligence and Humanized Computing*.

[8] Ward R., Sreenivas S., Read J., Saunders K. E. A., Rogers R. D. (2017). The role of serotonin in personality inference: tryptophan depletion impairs the identification of neuroticism in the face. *Psychopharmacology*.

[9] Dembani R., Zheng W., Sun M., Uddin N. (2020). Unsupervised facial expression detection using genetic algorithm. *Neural Network World*.

[10] Li W. (2021). Design of smart campus management system based on internet of things technology. *Journal of Intelligent and Fuzzy Systems*.

[11] Rahman S. M. M., Howlader T., Hatzinakos D. (2016). On the selection of 2D Krawtchouk moments for face recognition. *Pattern Recognition*.

[12] Zhang J., Deng Y., Guo Z., Chen Y. (2016). Face recognition using part-based dense sampling local features. *Neurocomputing*.

[13] Cho M., Jeong Y. (2017). Face recognition performance comparison between fake faces and live faces. *Soft Computing*.

[14] Özyurt Ö., Özyurt H. (2016). Using Facebook to enhance learning experiences of students in computer programming at Introduction to Programming and Algorithm course. *Computer Applications in Engineering Education*.

[15] Yin X., Liu X. (2018). Multi-Task convolutional neural network for pose-invariant face recognition. *IEEE Transactions on Image Processing*.

[16] Chong L. Y., Ong T. S., Teoh A. B. J. (2019). Feature fusions for 2.5D face recognition in random maxout extreme learning machine. *Applied Soft Computing*.

[17] Yang W., Wang Z., Zhang B. (2016). Face recognition using adaptive local ternary patterns method. *Neurocomputing*.

[18] Long B., Yu K., Qin J. (2017). Data augmentation for unbalanced face recognition training sets. *Neurocomputing*.

[19] Becerra-Riera F., A Morales-González H., Méndez-Vázquez. (2017). Facial marks for improving face recognition. *Pattern Recognition Letters*.

[20] Hao K. (2020). Multimedia English teaching analysis based on deep learning speech enhancement algorithm and robust expression positioning. *Journal of Intelligent and Fuzzy Systems*.

[21] Shao W. Y., Guo Y. F. (2016). Application of multi task learning and convolutional neural network in face recognition. *Computer engineering and application*.

[22] Feng J. Y., Chen H. Y. (2017). Research on face recognition based on artificial neural network. *Automation and instrumentation*.

[23] Han S., Ren F., Wu C., Chen Y., Du Q., Ye X. (2018). Using the tensorflow deep neural network to classify mainland China visitor behaviours in Hong Kong from check-in data. *ISPRS International Journal of Geo-Information*.

[24] Qi Y. Q., Wang L. J., Wu S. W. (2016). A face recognition algorithm based on sparse representation and neural network. *Computer applications and software*.

[25] Li N., Cai J. Y., Li K. (2020). Face recognition algorithm based on convolutional neural network with multi perception structure. *Computer system applications*.

[26] Xuan H., Zhong W. F., Chen W. (2018). Application of face recognition technology in teaching management of Tsinghua University. *China education informatization*.

[27] Yan Y. Y., Guo H. L. (2018). Application of face recognition system based on convolutional neural network in teaching management. *China educational technology equipment*.

[28] Zhang H., Liu B., Wang F. (2019). Research on the application of face recognition technology in university educational administration. *China education informatization*.

[29] Liu C. F., Liang F. Q. (2018). Research and application of face recognition technology in student status management system. *Journal of Chifeng University: Natural Science Edition*.

[30] Yao S. (2020). Architecture design of student behavior management system based on face recognition technology. *Electronic technology and software engineering*.

[31] Deng W., Shang S., Cai X. (2021). Quantum differential evolution with cooperative coevolution framework and hybrid mutation strategy for large scale optimization. *Knowledge-Based Systems*.

[32] Zielonka A., Sikora A., Woźniak M. (2020). Intelligent Internet of things system for smart home optimal convection. *IEEE Transactions on Industrial Informatics*.

[33] Cui K., Jing X. (2019). Research on prediction model of geotechnical parameters based on BP neural network. *Neural Computing & Applications*.

[34] Han Y., Liu C., Yan L., Ren L. (2021). Design of decision tree structure with improved BPNN nodes for high-accuracy locomotion mode recognition using a single IMU. *Sensors*.

[35] Cai X., Zhao H., Shang S. (2021). An improved quantum-inspired cooperative co-evolution algorithm with muli-strategy and its application. *Expert Systems with Applications*.

[36] Kumari N., Bhatt A., Dwivedi R., Belwal R. (2021). Hybridized approach of image segmentation in classification of fruit mango using BPNN and discriminant analyzer. *Multimedia Tools and Applications*.

[37] Cui K., Qin X. (2018). Virtual reality research of the dynamic characteristics of soft soil under metro vibration loads based on BP neural networks. *Neural Computing & Applications*.

